# Bioinformatics Analysis Reveals *MCM3* as an Important Prognostic Marker in Cervical Cancer

**DOI:** 10.1155/2021/8494260

**Published:** 2021-10-11

**Authors:** Hui Ma, Zhen Liu, Honglin Li, Xuewang Guo, Sujie Guo, Pengpeng Qu, Yuquan Wang

**Affiliations:** ^1^Department of Gynecology, The Secondary Hospital of Tianjin Medical University, No. 23 Pingjiang Road, Hexi District, Tianjin 300211, China; ^2^Department of Gynecology, Chifeng Municipal Hospital, Chifeng Clinical Medical School of Inner Mongolia Medical University, Chifeng 024099, China; ^3^Department of Gynecology Oncology, Tianjin Central Hospital of Gynecology & Obstetrics, 156 Sanmalu, Nankai, Tianjin 300100, China

## Abstract

The minichromosome maintenance complex 3 (MCM3) is essential for the regulation of DNA replication and cell cycle progression. However, the expression and prognostic values of MCM3 in cervical cancer (CC) have not been well-studied. Herein, we investigated the expression patterns and survival data of MCM3 in cervical cancer patients from the ONCOMINE, GEPIA, Human Protein Atlas, UALCAN, Kaplan-Meier Plotter, and LinkedOmics databases. The expression level of MCM3 is negatively correlated with advanced tumor stage and metastatic status. Specifically, MCM3 is significantly differentially expressed between patients in stage 1 and stage 3 cervical cancer with *p* value 0.0138. Similarly, the *p* values between stage 1 and stage 4 cervical cancer, between stage 2 and stage 3, and between stage 2 and stage 4 are 0.00089, 0.0244, and 0.00197, respectively. Not only that, cervical cancer patients with high mRNA expression of MCM3 may indicate longer overall survival but indicate shorter relapse-free survival. PRIM2 and MCM6 are positively correlated genes of MCM3. Bioinformatics analysis revealed that MCM3 might be considered a biological indicator for prognostic evaluation of cervical cancer. However, it is currently limited to bioinformatics analysis, and more clinical tissue specimens and cell experiments are needed to further explore the role of MCM3 in the occurrence and progression of cervical cancer.

## 1. Introduction

Cervical cancer is a common gynecological tumor. The incidence rate and mortality rate rank fourth in the female malignant tumor worldwide, only behind breast, colorectal, and lung cancer [1]. However, in developing countries, the incidence and mortality of cervical cancer rank second only to breast cancer in female malignant tumors [2]. Cervical cancer is one of the cancers that can be prevented through screening. With the widespread popularity of screening, the incidence of cervical cancer is declining year by year. However, as early cervical cancer has no symptoms, many patients are already in the middle and advanced stages of disease when they were diagnosed [3]. The main treatments for cervical cancer include surgery, radiotherapy, and adjuvant platinum-based chemotherapy. Early cervical cancer is mainly treated by surgery, and the 5-year survival rate can reach 88-95%. However, there are limited treatment methods for patients in the middle and advanced stages, and the therapeutic effect of radiotherapy and chemotherapy is not satisfactory [4–6]. Therefore, it is urgently needed to discover novel molecular biomarkers, therapeutic targets, or prognostic evaluation index for cervical cancer. The extensive application of bioinformatics databases has facilitated the discovery of new biomarkers for cancer management [7–10].

The minichromosome maintenance complex (MCM) family proteins (MCM2–8 and MCM10) play an essential role in the initiation of the DNA replication process and cell division [11, 12]. MCM2-7 complex acts as a helicase during the initiation of DNA replication while MCM8 performs a similar uncoiling effect during the elongation of DNA replication. In addition, MCM10 participates in the regulation of DNA replication elongation [13, 14]. MCM3 is one of the MCM families. MCM3 acetylation could initiate DNA replication and cell cycle progression [15]. MCM3 expression is upregulated in a variety of malignant tumor cells [16]. Moreover, the expression of MCM3 is deregulated in several human malignancies, including lung cancer [17], colorectal cancer [18], liver cancer [19], breast cancer [20], ovarian cancer [21], and oral squamous cell carcinoma [22]. Zhou et al. found that colorectal cancer patients with high expression of MCM3 have a poor prognosis [18]. A study of liver cancer showed that high expression of MCM3 was associated with tumor invasion and poor prognosis of liver cancer patients [19]. Løkkegaard et al. found that ER+ breast cancer cells can develop resistance to tamoxifen and letrozole by upregulating MCM3 [20].

Despite the intensive study of MCM3 in many cancers, there is limited research regarding MCM3 in cervical cancer. By studying the role of MCM3 in cervical cancer, it might provide a novel biomarker for drug development and repositioning on this cancer.

## 2. Methods

### 2.1. ONCOMINE Analysis

ONCOMINE (https://www.oncomine. org/resource/login.html) is an online bioinformatics database [23]. In this study, we used ONCOMINE to analyze the transcription levels of MCM3 mRNA and compare the expression of MCM3 in cervical cancer and normal cervical tissues, Shan parameters: *p* < IE − 4, fold change > 2, and gene rank: 10%.

### 2.2. GEPIA Dataset

GEPIA (http://gepia.cancer-pku.cn/) is an interactive web server for analyzing the RNA sequencing expression data from TCGA and GTEx projects [24, 25]. We used GEPIA to compare the expression of MCM3 mRNA in cervical tumor/normal tissues. The differences in transcription expression was determined by Student's *t*-test, and *p* values < 0.05 were considered statistically significant.

### 2.3. TIMER 2

TIMER (https://cistrome.shinyapps.io/timer/) is a comprehensive resource for the systematic analysis of immune infiltrates [26]. We used TIMER to analyze the correlation between the expression of MCM3 in cervical cancer and the abundance of the six immune infiltrates, including B cells, CD4+ T cells, CD8+ T cells, neutrophils, macrophages, and dendritic cells in cervical cancer. The scatterplots show purity-corrected partial Spearman's rho.

### 2.4. Human Protein Atlas

The Human Protein Atlas (https://www.proteinatlas.org/) is aimed at mapping all the human protein in cells, tissues, and organs, including antibody-based imaging [27]. We use this database to retrieve immunohistochemical staining pictures of MCM3 in cervical cancer and normal cervix.

### 2.5. Kaplan-Meier Plotter

Kaplan-Meier Plotter (https://kmplot.com/analysis/) is a large sample-based dataset that is able to evaluate the survival of patients with different types of cancers [28]. We used the Kaplan-Meier Plotter to analyze the prognostic value of MCM3 expression in cervical cancer. *p* < 0.05 was considered statistically significant. The hazard ratios (HRs) with specific 95% confidence intervals (CIs) and *p* values were listed.

### 2.6. UALCAN Cancer Database

UALCAN (http://ualcan.path.uab.edu/) uses data from the Clinical Proteomic Tumor Analysis Consortium (CPTAC) Confirmatory/Discovery dataset to provide protein expression analysis option [29]. We evaluated the expression of MCM3 in cervical cancer by TCGA analysis.

### 2.7. LinkedOmics Dataset

LinkedOmics (http://www.linkedomics.orglogin.php) is a new and unique datasets for disseminating data from large-scale cancer omics projects [30]. We used this database to find genes closely related to MCM3.

## 3. Results

### 3.1. MCM3 Expression Level across Cancers

We used the ONCOMINE database to compare the expression levels of MCM3 mRNA across cancers and its mRNA expression with that in corresponding normal tissues.  Figure 1(a) presents the expression of the MCM3 across cancers. The results showed that MCM3 expression was higher in several cancer groups than in normal tissues, including the bladder, brain, breast, cervical, colorectal, liver, head and neck, and lung, as well as lymphoma. However, the mRNA expression of MCM3 was significantly downregulated in leukemia and brain cancers. Moreover, we further used TIMER to evaluate the expression of MCM3 in TCGA.  Figure 1(b) shows the details of MCM3 expression across cancers.

### 3.2. Overexpression of MCM3 in Cervical Cancer

ONCOMINE and GEPIA datasets were used to compare the expression level of MCM3 in cervical cancer with those in corresponding normal tissues. We further used the Human Protein Atlas database to retrieve immunohistochemical staining pictures of MCM3 in cervical tissues.  Figure 2(a) presents the expression of the MCM3 in cervical cancer compared with normal tissues. MCM3 were significantly upregulated in cervical cancer tissues. The details are shown in Table 1 [25, 31, 32]. In addition, we compared the MCM3 protein expression level in cervical cancer and normal cervical tissues through the Human Protein Atlas datasets (Figure 2(b)).

### 3.3. Relationship between the Expression Levels of MCM3 mRNA and the Clinicopathological Parameters of Patients with Cervical Cancer

We used the GEPIA dataset and UALCAN cancer database to analyzed clinicopathological parameters for cervical cancer. MCM3 expression was significantly related to tumor stage (Figure 3(a), *p* < 0.001) and lymph node metastasis (Figure 3(b), *p* < 0.001), whereas age (Figure 3(c), *p* > 0.05), race (Figure 3(d), *p* > 0.05), weight (Figure 2(e), *p* > 0.05), tumor histology (Figure 3(f), *p* > 0.05), and tumor grade (Figure 3(g), *p* > 0.05) were not significantly associated. We further analyzed the prognostic value of MCM3 in cervical cancers in the Kaplan-Meier Plotter. The detailed results are shown in Figure 3(h). The Kaplan-Meier curve and log rank test analyses revealed that the increased MCM3 mRNA levels were significantly associated with better overall survival (OS) (*p* < 0.05) of all of the patients with cervical cancer. On the contrary, increased MCM3 mRNA levels were significantly associated with shorter relapse-free survival (RFS) (*p* < 0.05).

### 3.4. Correlations between MCM3 Expression and Immune Infiltration in CC

Immune infiltration in the tumor microenvironment can affect the survival of patients. Next, we analyzed the correlation between the expression of MCM3 in cervical cancer and immune infiltration. Cervical cancer patients had good survival with high MCM3 expression. We used the TIMER database to explore the correlation between MCM3 and immune cell infiltration in cervical cancer. The results showed that MCM3 was significantly related to the purity of cervical cancer (*R* = 0.128, *p* = 3.23*e* − 02). The expression of MCM3 was significantly positively correlated with the infiltration level of CD4+ T cells (*R* = 0.133, *p* = 2.66*e* − 02), neutrophils (*R* = 0.137, *p* = 2.23*e* − 02), B cells (*R* = 0.214, *p* = 3.31*e* − 04), and CD8+ T cells (*R* = 0.127, *p* = 3.45*e* − 02), while the expression of MCM3 was significantly negatively correlated with the infiltration level of macrophages (*R* = −0.201, *p* = 7.67*e* − 04) and dendritic cells (*R* = −0.208, *p* = 4.91*e* − 04) in cervical cancers (Figure 4).

### 3.5. Correlation Analysis

In order to further study the potential mechanism of MCM3 in cervical cancer, we excavated the gene data coexpressed with MCM3 by the GEPIA database and LinkedOmics database. PRIM2 is a correlated gene (Figures 5(a) and 5(b), Table 2). Further analysis using the GEPIA database and LinkedOmics database revealed the correlation between MCM3 and PRIM2 or MCM6. Pearson correlation analysis showed that the expression of MCM3 and PRIM2 or MCM6 in cervical cancer was obviously positive (*R* = 0.6387 and *R* = 0.5443, respectively, Figures 5(c) and 5(d)).

PRIM2 and MCM6 were significantly upregulated in cervical cancer tissues by the GEPIA database (Figures 6(a) and 6(d)). We further used the Kaplan–Meier plotter database to analyze the survival of cervical cancer patients, and the analysis results suggest that the upregulation of PRIM2 and MCM6 is related to the longer OS of cervical cancer patients (Figures 6(b) and 6(e)), while only MCM6 is related to shorter RFS, which is similar to MCM3.

## 4. Discussion

Previous studies have shown overexpression of MCM3 in many cancers [15–18, 20, 21]. Zhou et al. [18] found that elevated MCM3 expression was associated with poor prognosis of CRC patients. They further confirmed that MCM3 was overexpressed in CRC cell lines through vitro experiments. In addition, knockdown of MCM3 in CRC cells could significantly inhibit CRC cell proliferation, migration, invasion, and transition of the G1 to S phase. Decreasing the expression of MCM3 in endocrine-resistant cells restored drug sensitivity, and detecting the expression of MCM3 may predict the response of patients to endocrine treatment [20]. Another study in ovarian cancer showed that increased expression of MCM-3 and Ki-67 was associated with increased histological malignancy [21]. Compared with controls, MCM3 were highly expressed in CSCC, and MCM3 expression was correlated with CSCC cell differentiation, while, in terms of prognostic value assessment, there is no independent prognostic correlation between MCM3 and clinicopathological parameters [33]. Although the role of MCM3 in the tumorigenesis and prognosis of several cancers has been partially confirmed, further bioinformatics analysis of cervical cancer has yet to be performed. Importantly, the current study focuses on the analysis of exploring the expression and prognostic values of MCM3 in cervical cancer. We hope that the current findings will contribute to provide new ideas for the clinical diagnosis, prognosis assessment, and targeted therapy of cervical cancer. In our study, ONCOMINE datasets and the GEPIA database revealed that the expression of MCM3 was significantly higher in cervical cancer than in normal tissues. MCM3 expression was significantly related to tumor stage (*p* < 0.001) and lymph node metastasis (*p* < 0.001). A high MCM3 expression was significantly associated with better OS in patients with cervical cancer.

The tumor microenvironment (TME) could affect the progression and recurrence of tumors and has received increasing attention. Immune cells are considered an important determinant of clinical outcome and immunotherapy response [34]. Our study shows that the expression of MCM3 may be significantly related to the infiltration of six immune cell types, indicating that MCM3 may also reflect the immune status in addition to the prognosis of the disease. This research may provide detailed immune information to help design new immunotherapies.

We further searched genes closely related to MCM3 through the GEPIA database, UALCAN cancer database, and LinkedOmics. We selected two proteins PRIM2 and MCM6, which have strong correlation with MCM3 and have different expressions in cervical cancer compared with normal cervical tissues. Through analysis, we found that the expression of PRIM2 and MCM6 was positively correlated with MCM3 expression. We further evaluate their prognostic value in cervical cancer.

PRIM2 is a large subunit of DNA primase, located at 6p11.1–p12 of the human chromosome [35, 36]. The upregulated expression of PRIM2 in cervical cancer enhanced DNA synthesis, accelerated the progression of cell cycle from the G1 to S phase, and promoted the proliferation of cervical cancer cells and the growth of cervical cancer [37]. MCM6 is a number of the minichromosome maintenance complex (MCM) family proteins [11, 13]. In a study of lung cancer [38], the high expression of MCM6 suggests a short overall survival. However, contrary to the conclusions of this study, we found that patients with high expression of MCM6 have a better overall survival but have a poor disease progression-free survival.

In summary, this analysis shows that MCM3 is more highly expressed in cervical cancer than normal cervical tissues. The results indicate that MCM3, PRIM2, and MCM6 could be used for early detection of cervical cancer and may be used as indicators of prognosis. Moreover, MCM3 may become the target of immunotherapy for cervical cancer in the future.

However, our current research has some limitations. All the data analyzed in this study are from bioinformatics databases. We will further explore the potential mechanism of MCM3 in cervical cancer by clinical tissues and cervical cancer cell lines in in vivo and in vitro experiments.

## Figures and Tables

**Figure 1:** MCM3 expression levels across cancers. (a) The transcription levels of MCM3 across cancers. The figure is generated from ONCOMINE with exact thresholds (*p* value: IE-4; fold change: 2; gene rank: top 10%). (b) MCM3 expression levels across cancers from TCGA data in TIMER 2. ^∗^*p* < 0.05, ^∗∗^*p* < 0.01, and ^∗∗∗^*p* < 0.001.

**Figure 2:** The expression of MCM3 in cervical cancer: (a) GEPIA box plot; (b) IHC of MCM3 in normal (N) and tumor (T) tissues from patients with cervic al cancer in the Human Protein Atlas.

**Figure 3:** Box plot revealing the relationship between MCM3 expression and different clinical indicators using the UALCAN cancer database shown for stage (a), nodal metastasis (b), age (c), race (d), weight (e), tumor histology (f), and tumor grade (g); analysis is shown for OS (h) and RFS (i) by the Kaplan–Meier Plotter.

**Figure 4:** The correlation between MCM3 expression and immune infiltration level in CC. Correlation of MCM3 expression with tumor purity and infiltrating levels of B cell, CD8+ T cell, CD4+ T cell, macrophage, neutrophil, and dendritic cell in CC. *p* < 0.05 is considered statistically significant. CC: cervical cancer.

**Figure 5:** Coexpression analysis of MCM3: (a, b) coexpression profile of MCM3 identified using the LinkedOmics dataset; (c) the correlation between MCM3 and PRIM2 expression in cervical cancer by the LinkedOmics dataset; (d) the correlation between MCM3 and MCM6 expression in cervical cancer by the LinkedOmics dataset.

**Figure 6:** PRIM2 and MCM6 in cervical cancer: (a) the expression of PRIM2 showed by the GEPIA database; (b) the OS status for the expression of PRIM2 from the Kaplan–Meier Plotter; (c) the RFS status for the expression of PRIM2 from the Kaplan–Meier Plotter; (d) the expression of MCM6 showed by the GEPIA database; (e) the OS status for the expression of MCM6 from the Kaplan–Meier Plotter; (f) the RFS status for the expression of MCM6 from the Kaplan–Meier Plotter.

**Table 1:** Datasets of MCM3 expression in cervical cancers (ONCOMINE database).

Cancer site	Types of cancer vs. normal	Fold change	*t*-test	*p* value	Dataset
MCM3	Cervical cancer vs. normal	4.180	11.188	2.84*E*-13	Pyeon
	Cervical squamous cell carcinoma vs. normal	2.613	7.947	1.05*E*-10	Scotto
	Cervical squamous cell carcinoma vs. normal	2.589	12.088	1.48*E*-6	Biewenga

**Table 2:** Coexpression profile of MCM3 identified using the GEPIA database.

Gene symbol	Gene ID	PCC
PRIM2	ENSG00000146143.17	0.75
MCM6	ENSG00000076003.4	0.69
MUT	ENSG00000146085.7	0.68
CENPQ	ENSG00000031691.6	0.66
TIMELESS	ENSG00000111602.11	0.65
DEK	ENSG00000124795.14	0.65
SRSF3	ENSG00000112081.16	0.64
TJAP1	ENSG00000137221.14	0.63
TXNDC16	ENSG00000087301.8	0.63
RBMX	ENSG00000147274.14	0.63

## Data Availability

The data used in this study was downloaded from TCGA website under the selection of cervical cancer (https://portal.gdc.cancer.gov/).
